The article "Control of hybrid electromagnetic bearing and elastic foil gas bearing under deep learning" was retracted in 2025. Reasons: compromised peer review; unreliable results or conclusions; concerns about the peer review.

# Control of hybrid electromagnetic bearing and elastic foil gas bearing under deep learning

**DOI:** 10.1371/journal.pone.0243107

**Published:** 2020-12-02

**Authors:** Xiangxi Du, Yanhua Sun

**Affiliations:** School of Mechanical Engineering, Xi'an Jiao Tong University, Xi'an City 710049, China; University College London, UNITED KINGDOM

## Abstract

The hybrid electromagnetic and elastic foil gas bearing is explored based on the radial basis function (RBF) neural network in this study so as to improve its stabilization in work. The related principles and structure of hybrid electromagnetic and elastic foil gas bearings is introduced firstly. Then, the proportional, integral, and derivative (PID) bearing controller is introduced and improved into two controllers: IPD and CPID. The controllers and hybrid bearing system are controlled based on the RBF neural network based on deep learning. The characteristics of the hybrid bearing system are explored at the end of this study, and the control simulation research is developed based on the Simulink simulation platform. The effects of the PID, IPD, and CIPD controllers based on the RBF neural network are compared, and they are also compared based on the traditional particle swarm optimization (PSO). The results show that the thickness, spread angle, and rotation speed of the elastic foil have great impacts on the bearing system. The proposed CIPD bearing control method based on RBF neural network has the shortest response time and the best control effect. The controller parameter tuning optimization starts to converge after one generation, which is the fastest iteration. It proves that RBF neural network control based on deep learning has high feasibility in hybrid bearing system. Therefore, the results provide an important reference for the application of deep learning in rotating machinery.

## 1. Introduction

The level of industrialization is improving continually, and rotating machinery is also developing in a more excellent direction. In recent years, the emergence of electromagnetic bearings and gas bearings has made rotating machinery more and more efficient, and various advantages of these two bearings have made their applications more and more widespread [1–3]. Electromagnetic bearing is easy to be controlled, but there are many limitations for its application. Gas bearing has strong adaptability, but it is difficult to be controlled. Therefore, they are combined in this article to obtain a hybrid bearing system that integrates the advantages of both. At present, there are not many researches on hybrid bearings. Because reliability of the bearing is the first principle of its application, control research on it is essential first of all.

The control of bearing system is a kind of complex nonlinear problem. In recent years, the rise of deep learning has provided a good solution to this kind of problem, and scholars in various countries have researched it. Of which, there are many studies on the control of electromagnetic bearing targeting at rotor control and optimization [4–6]. Reddy et al. (2018) proposed a self-designed fuzzy logic controller based on an adaptive multi-population genetic algorithm to control active electromagnetic bearing [7]. Dhyani et al. (2018) applied a fuzzy PID controller based on moth flame optimization (MFO) to achieve optimal control of the active bearing system [8]. Nowadays, development of deep learning makes people use neural networks to achieve system optimization control when facing some nonlinear problems [9]. Mehrnoush et al. (2018) corrected the PID controller based on the fuzzy wavelet neural network model [10]. Ramachandran et al. (2018) used a PID controller based on the generalized Hopfield neural network to control the load frequency of the power system [11]. Thus, it proves that neural networks based on deep learning have outstanding control capabilities for nonlinear problems.

To sum up, the RBF neural network based on deep learning is used to adjust and control the PID bearing controller and the hybrid bearing system to optimize the control of the hybrid electromagnetic and elastic foil gas bearing, which can provide the theoretical basis and corresponding reference for control application of neural network in the bearing system.

## 2. Methodology

### 2.1 Hybrid electromagnetic and elastic foil gas bearing

Electromagnetic bearing generally is composed of two parts, covering the electrical equipment and mechanical structure [12]. Electromagnetic bearing is basically a combination of rotor and axial and radial electromagnetic bearing. It can generate electromagnetic force through current, and has a certain effect on the magnet material to enable the rotor to achieve contactless suspension [13]. The electromagnetic bearing and its working principle are shown in Fig 1.

**Fig 1:** Schematic diagram of electromagnetic bearing and its working principle.

As shown in Fig 1, the electromagnets are symmetrically fixed, and the rotor is placed between the electromagnets. If there is no external force, the relative electromagnetic force generated by the two electromagnets is the same after energization, and the rotor will be suspended in the air, without any touch to the inner wall of the bearing [14]. The displacement state of the rotor is monitored by a monitoring probe, and the displacement signal is transmitted to the controller. After calculation by the algorithm, the result is reflected to the electromagnetic device, and the power is adjusted according to the signal analysis [15]. As a result, the rotor can be stably suspended in the target area.

The elastic foil gas bearing is a self-acting dynamic pressure bearing taking gas as a lubricant, and the elastic foil has good adaptability [16]. When it works, the elastic foil can be adjusted according to the working environment and properties, thereby reducing the pressure fluctuation of the gas film [17]. The interaction force between the various parts of the foil support structure can consume the excess energy in the bearing, so that the bearing has better stability. The elastic foil gas bearing is shown in Fig 2 below.

**Fig 2:** Schematic diagram of elastic foil gas bearing and its entity.

The elastic foil gas bearing does not require corresponding lubrication and cooling, so it has a lower maintenance cost. Compared with traditional bearings, it is featured with relatively fast rotating speed, high accuracy, low power, little pollution, and long service life. In addition, it can run well in some harsh environments. Thus, it can be applied widely and extensively.

Electromagnetic bearing and elastic foil gas bearing are currently two typical high-speed support methods, with their own unique advantages. The state of the electromagnetic bearing can be controlled accordingly, but its carrying capacity is somewhat not good enough due to limitation from the material. The elastic foil gas bearing can work for a long time under various extreme environments, but the start and stop of the rotor cause excessive friction between the foil and the bearing, which may cause the foil to fall off, and the service life will be affected. Hybrid electromagnetic and elastic foil gas bearing can combine the advantages of them, so that it not only can improve the performance of the bearing, but also can increase the bearing capacity [18]. Its structure is shown in Fig 3.

**Fig 3:** Structure of hybrid bearing.

Combining the two types of bearings can realize the load distribution. When the electromagnetic bearing stops working in a sudden situation, the gas bearing can also take on the system operation requirements [19]. Therefore, the hybrid electromagnetic and elastic foil gas bearing is the most ideal support method in high-speed rotating machines.

### 2.2 Proportional, integral, and derivative bearing controller

The most frequently used controller for linear control is PID controller, which is also the earliest one used in bearing control. In simple terms, the algorithm principle of the PID controller is to use the linear combination of the proportion of the output deviation (P), the corresponding integral (I), and the derivative (D) as the controller's output [20]. The P of PID can reflect the signal error in time, the D will become larger when the P is small, and its response speed will also be affected. However, if the proportional coefficient is too large, the system can’t operate stably. I is usually used to remove the static error, which can improve the stability of the system. The differential link can reflect the change of the deviation and speed up the response speed of the system, but the system will lose stability if the differential coefficient is too large [21]. The control process of traditional PID controller is shown in Fig 4.

**Fig 4:** The control process of traditional PID controller.

The mathematical model of the PID controller is shown in Eq (1).

$$S\left(t\right)=K_{p}e\left(t\right)+K_{i}\int_{0}^{t}e\left(t\right)+K_{d}\frac{de\left(t\right)}{dt}$$ (1)

In the above Eq (1), the output of the controller is represented by *S(t)*; the input is represented by *e(t)*; the proportional coefficient is represented by *K*_*p*_; the integral coefficient is represented by *K*_*i*_; and the differential coefficient is represented by *K*_*d*_.

The commonly used PID controllers are relatively simple and have stable control, the parameters are relatively easy to be adjusted, and there is no static error [22]. If the control object is a system that changes continuously over time, the parameters of the PID controller are not easy to be automatically adjusted to meet the control requirements of the system, and the corresponding control effect is not very ideal [23]. Therefore, the traditional PID controller needs to be modified to improve its control performance. For other bearings with hybrid electromagnetic and elastic foil, stable load-bearing requires a certain eccentric force between the bearing and the journal. However, the center of gravity of the electromagnetic bearing in the traditional PID controller coincides with the journal, so it is necessary to distribute the load in the hybrid bearing by other means to solve the above problems, thereby improving the overall carrying capacity of the hybrid bearing.

The traditional PID controller is modified in this article. In the traditional algorithm, if the rotor shifts suddenly and the immediate shift is small, the value of its derivative term will still become very large, which will also increase the control signal. The adjusted PID output is shown in Eq (2).

$$s_{IPD}\left(t\right)={-K}_{p}g_{m}\left(t\right)+K_{i}\int_{0}^{t}e\left(t\right)-\frac{dg_{m}\left(t\right)}{dt}$$ (2)

As shown in above Eq (2), the value of the derivative term of the PID controller after adjustment will not be affected by the error, but will respond according to the value obtained by the feedback. This improved PID controller only retains the integral term, which is recorded as IPD control. g_m_(t) refers to the output after adjustment.

Another improvement way is to connect P D and P I in series, thereby obtaining a series PID controller, denoted as cascaded proportional-integral-derivative controller (CPID). Its output is shown in Eq (3).

$$s_{CPID}\left(t\right)=K_{p}^{C}\left(e\left(t\right)+K_{d}^{C}\frac{de\left(t\right)}{dt}\right)+K_{i}^{C}\int_{0}^{t}\left(e\left(t\right)+K_{d}^{C}\frac{de\left(t\right)}{dt}\right)dt$$ (3)

In the above Eq (3), the proportional coefficient after series is represented by *K*^*c*^_*p*_; the integral coefficient is represented by *K*^*c*^_*i*_; and the differential coefficient is expressed in terms of *K*^*c*^_*d*_.

### 2.3 Bearing control method based on deep learning

Deep learning is a feature learning method undertaking neural network as the basic structure of learning. Deep learning provides a better way to solve some complex problems [24]. As the basis of deep learning, artificial neural network (ANN) has the ability to adapt to the characteristics of autonomous learning of complex problems and can deal with nonlinear problems well [25]. RBF neural network has good generalization ability and can approach nonlinear problems with unlimited accuracy [26–28]. But when there is not enough data, the neural network can’t function normally. To achieve the control optimization, there are strict requirements on the mathematical model of the system, which is the same as the PID controller [29]. The hybrid electromagnetic and elastic foil gas bearing system itself is nonlinear, the corresponding parameters are not certain enough, and it is not easy to achieve the precise control. Therefore, it is necessary to combine the PID controller with the neural network algorithm and the improvement has to be made to solve the control difficulties to the maximal degree [30].

The RBF neural network can learn and map according to the local information, so as to achieve the data collection and parameters self-adjustment. The structure of RBF neural network is similar to that of the human brain, and it also has similarities during the work. The change of local information and the receiving interval of neurons overlap with the brain and nervous system, and gradually approach the whole from the local. This also shows that the RBF neural network can gradually approximate any nonlinear function in the calculation operation with any given accuracy. The basic structure of RBF neural network is illustrated in Fig 5 below.

**Fig 5:** Basic structure of radial basis function neural network.

The approximation characteristics of the RBF neural network make each neuron in its hidden layer represents a result of this local approximation, and its weighted summation is used to replace the local approximation of the hidden layer with an overall approximation.

The mapping function of the hidden layer is shown in Eq (4).

$$g_{a}\left(x\right)=f_{a}\left(\frac{\left\|X-C_{a}\right\|}{b_{a}}\right),a=1,2,\cdots ,P$$ (4)

The central vector expression of the node in the *a*^*th*^ hidden layer can be expressed as below.

$$C_{a}={\left[C_{a1},C_{a2},\cdots ,C_{ak},\cdots {,C}_{aN}\right]}^{T}\left(k=1,2,\cdots ,N\right)$$ (5)

In the above Eqs (4) and (5), *g*_*a*_*(x)* refers to the output in hidden layer, and *X* indicates the specified output value. It is assumed that the basis width vector of the RBF neural network is represented by *b*, then *b*_*a*_ represents the base width vector of node *a*. The size of this parameter can be chosen randomly, but it has to be greater than 0. Its function is to determine the width of the basis function around its center. *f*_*a*_ represents a radially symmetric function with only one maximal value at *C*_*a*_.

Mapping equation of the output layer can be expressed as below.

$$h_{1}\left(x\right)=g_{1}w_{1}+g_{2}w_{2}+\cdots +g_{P}w_{P}$$ (6)

In the above Eq (6), the output weight vector is represented by *w*.

The most commonly used radial basis function is the Gaussian function, and the function expression is shown in Eq (7):

$$g_{a}\left(x\right)=f_{a}\left(\frac{\left\|X-C_{a}\right\|}{b_{a}}\right)=\exp\left(-\frac{{\left\|X-C_{a}\right\|}^{2}}{b_{a}^{2}}\right)$$ (7)

It can be known from Eq (7) that the output interval range of the node is [0, 1], and the distance between the input sample and the output value to the center of the node is directly proportional. The RBF neural network has a larger response range as C increases, and the smoothness of each neuron function will also increase. If the value of *C* becomes smaller, the image of the function will show a prominent upper end, and the distance between the lower ends decreases, so that the function can only sensitively receive input close to the weight vector, which can cause serious impact to the overall control ability of the neural network.

A feedforward compensation and feedback control bearing system model is established based on the RBF neural system. It can adjust the rotor system and the PID controller synchronously, so that the control parameters can be adjusted accurately while reducing the response time, making the control system becomes faster, more accurate, and more effective. Feedback control can eliminate the deviation of the neural network when approaching the bearing system. The control idea of hybrid electromagnetic and elastic foil gas bearing based on RBF neural network and PID controller is shown in the Fig 6.

**Fig 6:** Control idea of hybrid bearing system.

Fig 6 suggests that the total output of the controller is the sum of the output of the PID controller and that of the RBF neural network, so it can be calculated with Eq (8).

$$P=P_{PID}+P_{RBF}$$ (8)

## 3. Results and discussion

### 3.1 Analysis result of hybrid bearing

A hybrid bearing system is obtained by combining the electromagnetic bearing and elastic foil gas bearing. In order to control the hybrid electromagnetic and gas bearing system, it has to analyze its characteristics firstly. In the actual operation of the bearing, the eccentricity of the bearing rotor will be automatically adjusted with the change of the rotor load when the rotation speed is fixed, thus achieving a stable state. The capacity and friction torque of the hybrid bearing system during operation are explored in terms of thickness, spread angle, and eccentricity and rotating speed of the hybrid bearing system to judge the overall performance of the hybrid bearing system. The influence of foil thickness on the bearing capacity of the hybrid bearing system under different eccentricities is illustrated in Fig 7.

**Fig 7:** Influence of foil thickness on the bearing capacity of the hybrid bearing system under different eccentricities.

When the eccentricity is small, the bearing capacity of the hybrid bearing system will increase as the thickness of the foil increases. Because the thicker the foil, the greater the rigidity of its support, so it can have a greater bearing capacity under the same eccentricity. When the eccentricity is relatively large, the bearing capacity of the hybrid bearing system will increase firstly and then slightly decrease as the thickness of the foil increases. This is because when the eccentricity is relatively large, the increase in the thickness of foil can increase the thickness of the gas film, the effective bearing area of the gas film decreases, and the bearing capacity of the bearing system decreases. Fig 7 indicates that when the foil thickness is about 0.12 mm, the hybrid bearing system can obtain the maximum bearing capacity under the condition of large eccentricity.

The influence of foil thickness on the friction torque of hybrid bearing system under different eccentricities is shown in Fig 8.

**Fig 8:** The influence of foil thickness on the friction torque of hybrid bearing system under different eccentricities.

According to Fig 8, it can be seen that the friction torque increases with the continuous increase of the thickness of the foil. When the thickness of the elastic foil increases, the rigidity of its support increases, resulting in a continuous decrease in the thickness of the gas film at the end of the foil. In addition, it is boundary of the atmosphere at the end of gas film, and its pressure gradient is relatively large, so the friction torque is large. In order for the hybrid bearing system to reduce the heat generation, it is necessary to select a relatively thin elastic foil while ensuring its bearing capacity.

The influence of the spread angle of the foil on the bearing capacity of the hybrid bearing system under different eccentricities is shown in Fig 9.

**Fig 9:** The influence of the spread angle of the foil on the bearing capacity under different eccentricities.

Under the condition that the eccentricity keeps increasing, the bearing capacity of the hybrid bearing system decreases firstly and then increases as the spread angle of the elastic foil increases. When the spread angle of the elastic foil continues to increase, its corresponding contact area increases. When the adjacent foils overlap, they can bear the pressure brought by the gas film together, thereby improving the bearing capacity of the hybrid bearing. The position with high pressure in the gas film is at the end of the foil, and supporting rigidity of the end can directly affect the pressure brought by the gas film. When the spread angle of the elastic foil continues to increase, the supporting rigidity of the foil end decreases firstly and then increases. Therefore, the combined effect of these factors causes first-increase and then-decrease in bearing capacity of the hybrid bearing system and in spread angle of the elastic foil.

The influence of foil spread angle on friction torque under different eccentricities is shown in Fig 10.

**Fig 10:** The influence of foil spread angle on friction torque under different eccentricities.

Fig 10 illustrates that when the eccentricity is relatively small, the friction torque decreases as the spread angle of the elastic foil increases. When the eccentricity is relatively large, the friction torque decreases firstly and then increases as the spread angle of the elastic foil increases. This is caused by changes in thickness and pressure of gas film.

The influence of eccentricity on the bearing capacity and friction torque of the hybrid bearing system at different rotating speeds is shown in Figs 11 and 12, respectively.

**Fig 11:** The influence of eccentricity on the capacity of the hybrid bearing system at different bearing rotating speeds.

**Fig 12:** The influence of eccentricity on the friction torque of the hybrid bearing system at different rotating speeds.

According to Figs 11 and 12, when the eccentricity increases, the bearing capacity and friction torque of the hybrid bearing system increase both. The higher the speed, the larger the bearing capacity and friction torque.

The analysis of hybrid electromagnetic and elastic foil gas bearing system proves that the results obtained in this study are similar to those obtained by Polyakov et al. (2019) [18]. There are many factors affecting the performance of hybrid bearing system. Thus, different bearing parameters should be formulated according to the requirements to obtain a better bearing system, so as to control its overall performance.

### 3.2 Control results of hybrid bearing

The hybrid electromagnetic and elastic foil gas bearing system has a more complicated structure, and the corresponding parameters can’t be determined. In order to control it better, it is necessary to select a control method for nonlinear problems. This article introduces the PID controller commonly used in the bearing systems, and has made corresponding improvements to it, so two improved controllers (IPD and CPID) are obtained. When using a controller, it can adjust its parameters automatically in order to adapt to the external conditions. However, the hybrid bearing system is a time-varying system, so it is difficult for the controller to automatically, so that the required control effect is hard to be achieved. An RBF neural network is proposed based on the deep learning method by combining the RBF neural network with the PID controller, which can not only realize the optimal control of the hybrid bearing system, but also make certain adaptive adjustments to the PID parameter setting. According to the characteristics of the infinite approximation of the RBF neural network, more precise control can be achieved, and the hybrid bearing system can operate more stably. Based on the Simulink simulation platform, this paper conducts simulation experiments on the PID feedback control of the hybrid bearing system combined with the RBF neural network. Thus, the simulation block diagram is given in Fig 13.

**Fig 13:** Simulation block diagram of hybrid bearing system control based on the RBF neural network.

For a better comparison and analysis, the optimization results of adaptive adjustment of controller parameters of the proposed RBF neural network control is compared with the traditional algorithm. The corresponding number of iterations is given in Fig 14.

**Fig 14:** Comparison on optimization results of controller with the RBF neural network and traditional algorithms.

Fig 14 reveals that, the RBF neural network control algorithm proposed has the fastest convergence speed compared with the traditional algorithm. In addition, RBF neural network combined with CPID controller can get the optimal solution after running for 1 generation, while the traditional algorithm starts to converge in the 13^th^ generation at the fastest. This result is similar to the research results of RBF neural network control algorithm in relevant literatures, which confirms the effectiveness of RBF neural network in bearing control research.

It compares the tracking response and tracking error of the three control methods to the hybrid bearing system, aiming to analyze the control effect of hybrid bearing system further, and the comparison results are shown in Fig 15.

**Fig 15:** Tracking response and tracking error of the three control methods to the hybrid bearing system.

It can be seen from Fig 15 that, the RBF neural network combined with the IPD controller has a greatly fluctuating tracking, and its tracking error fluctuations are also obvious. Relatively speaking, the RBF neural network combined with the CPID controller has the best control effect and relatively stable tracking. The research proves that the proposed RBF neural network combined with the feedback control of the controller has a better control effect on the hybrid bearing system.

## 4. Conclusion

In order to explore the control methods of the hybrid electromagnetic and elastic foil gas bearing system, an RBF neural network based on the deep learning method is proposed to control the PID controller and the hybrid bearing system. In this study, a simulation experiment is developed based on the Simulink simulation platform, and the controllers based on the RBF neural network are compared with those based on the traditional PSO. It is found that adjusting the structure of the hybrid electromagnetic and elastic foil gas bearing can obtain the best bearing system performance. When the hybrid bearing system is controlled by a PID controller, the PID controller can be controlled correspondingly with the aid of the RBF neural network control model. The experimental results prove that the RBF neural network control method based on the deep learning method has a better response effect in the control of the hybrid bearing system compared with the traditional PSO. This study has important reference value for the application of deep learning in the control of hybrid bearing system. However, there are still some shortcomings. It fails to improve the structure of the hybrid bearing. Future research can continue to optimize the structure of the hybrid bearing so that the system control can be more convenient.

## Supporting information

S1 File (XLSX)

S2 File (ZIP)
